This article has been retracted.

# MiR-199 Aggravates Doxorubicin-Induced Cardiotoxicity by Targeting TAF9b

**DOI:** 10.1155/2022/4364779

**Published:** 2022-07-15

**Authors:** Yangsheng Yu, Degang Guo, Lin Zhao

**Affiliations:** ^1^Department of Cardiology, Yantai Affiliated Hospital of Binzhou Medical University, Yantai, Shandong, China; ^2^Emergency Department, Third People's Hospital of Liaocheng City, Liaocheng 252000, China; ^3^Department of Cardiology, Sunshine Union Hospital of Weifang, Weifang 261000, Shandong, China

## Abstract

The clinical application of doxorubicin (DOX) is limited because of its cardiotoxicity. However, the pathogenic mechanism of DOX and the role of miRNA in DOX-induced cardiotoxicity remain to be further studied. This study aimed to investigate the role of miR-199 in DOX-mediated cardiotoxicity. A mouse model of myocardial cell injury induced by DOX was established. Quantitative real-time polymerase chain reaction (qRT-PCR) was used to detect the expression changes of miR-199 and TATA-binding protein associated factor 9B (TAF9b) in DOX-induced cardiac injury. Cell apoptosis was detected by TUNEL staining and flow cytometry. The expression levels of apoptosis-related proteins, namely, Bax and Bcl-2, were detected by qPCR. The expression of Beclin-1 and LC3b was detected by western blotting. The binding effect of miR-199 with TAF9b was verified by dual-luciferase reporter gene assay. In this study, overexpression of miR-199 could promote cardiotoxicity. Inhibition of miR-199 could alleviate DOX-mediated myocardial injury. Further studies showed that miR-199 targeted TAF9b. Moreover, miR-199 promoted apoptosis of myocardial cells and aggravated autophagy. Furthermore, we demonstrated that TAF9B knockdown reversed the myocardial protective effect of miR-199 inhibitors. Therefore, miR-199 promoted DOX-mediated cardiotoxicity by targeting TAF9b, thereby aggravating apoptosis and regulating autophagy.

## 1. Introduction

Doxorubicin (DOX) is an effective and commonly implemented anticancer drug for hematological diseases and solid tumors, and it is implemented as a first-line drug for a variety of cancers [1–3]. However, DOX can lead to multiple-organ toxicity in patients. As an anticancer agent, DOX can lead to long-term dose-dependent cardiotoxicity and heart failure [4, 5]. Mechanisms of DOX-mediated myocardial injury comprised cardiomyocyte abiosis [6], atrophy [7], autophagy disturbance [8], and oxidative stress [9].

The molecular mechanisms of DOX-induced cardiotoxicity have been extensively reported [10–13]. At present, free radicals produced by DOX are the primary cause of cardiotoxicity, involving nonenzymatic pathways mediated by Fe^3+^ and enzymatic pathways involved in antioxidant-related enzymes [14–17]. Thus, antioxidants prevent or mitigate cardiotoxicity induced by the elimination of excess free radicals produced by DOX.

MiRNAs are small noncoding RNAs that regulate the stability or translation of messenger RNA by interacting with specific sequences in the coding or untranslated regions to control gene expression. In recent years, its role in cardiovascular diseases has been slowly discovered, such as atherosclerosis [18,19], myocardial infarction [20], ischemia-reperfusion injury [21], and diabetic cardiomyopathy [22]. The mechanism of myocardial protection includes anti-apoptosis [23], inhibition of inflammation [21], and improvement of fibrosis to delay myocardial remodeling [22]. The role of miR-199 in DOX-mediated cardiomyopathy is included, particularly its effect on acute myocardial injury. Myocardial injury occurs in most patients after long-term administration of DOX [24, 25], but the role of miR-199 in cardiotoxicity mediated by DOX remains unknown.

TAF9b is a factor related to TATA-binding protein (TBP) [26]. TAF9b can bind to tumor suppressor proteins (p53). TAF9b participates in apoptosis by regulating p53 proteins [27, 28]. In previous studies, some scholars have proposed that TAF9b plays an indispensable role in transcriptional regulation [29]. Herein, we demonstrate that miR-199 aggravates apoptosis and regulates autophagy during DOX-mediated chronic cardiotoxicity by targeting TAF9b. It may be a new therapeutic target for cardiotoxicity mediated by oxidoreductase.

## 2. Materials and Methods

### 2.1. Animal Experiments

All the experiments were approved by the Animal Experimental Ethics Committee of Sunshine Union Hospital of Weifang. Eight-week-old female C57BL/6 mice were obtained from the Shanghai Model Organisms Center (Shanghai, China). C57BL/6 mice were raised in sterile filtration top cages with controlled humidity, a 12-hour day-night cycle, and a temperature of 22°C. Standard rodent food and tap water were provided randomly. Mice were intraperitoneally injected with Adriamycin (5 mg/kg; Sigma-Aldrich, St. Louis, USA, MO) weekly for 4 weeks, and then placed for 2 weeks to ensure complete absorption and effectiveness [30]. The mice were anesthetized with pentobarbital sodium (43 mg/kg iv) [31]. Blood and heart samples were collected at different time points to measure the changes of miR-199 under DOX stimulation. After the experiment, the mice were euthanized with CO_2_ and were put in a clean container. CO_2_ was injected at a rate of 20% per minute to replace the volume of the euthanasia box. After 10 minutes, make sure the mice are not moving, not breathing, and the pupils are dilated. Turn off CO_2_ and observe for another 2 minutes. The mice were confirmed to be completely dead.

### 2.2. HE Staining

Heart tissue was removed from a neutral formalin solution. After 24 h of running water washing, gradient alcohol dehydration was performed. Then, the tissue was dewaxed using xylene. After paraffin embedding, sectioning, xylene dewaxing, and staining for 15 min, sappan wood semen was washed with running water. After 30 s of blue infusion, the sample was rinsed with water for 15 min. Afterward, eosin staining and alcohol dehydration were performed. Finally, xylene and neutral resin sealing was conducted. The images were observed and collected under a light microscope (Nikon, Japan).

### 2.3. Cell Lines and Culture Conditions

The AC16 cell line was purchased from the American Type Culture Collection (ATCC, Manassas, VA, USA). The cells were cultured in a wet incubator containing 95% air and 5% CO_2_ at 37°C. The culture medium was Dulbecco's modified Eagle's medium (HyClone, USA) + 10% fetal bovine serum (Gibco, Life Technologies, Rockville, MA, USA). The culture medium was refreshed every 3 days, and when the cell density reached about 80%, the culture medium was replaced with serum-free DMEM for 12 h. Then, DOX (0.5 *μ*M) [30, 32–34] was implemented to induce cardiomyocyte injury.

### 2.4. Cell Transfection

MiR-199 mimics and inhibitors (Ribobio, China) were implemented to overexpress and downregulate miR-199 in vitro. We synthesized a small interfering RNA to knock out TAF9b (GenePharma, China). Random sequence molecules were synthesized as negative control. Control overexpression plasmids (100 nM), TAF9b overexpression plasmids (100 nM), were constructed by Shanghai GenePharma Co., Ltd. AC16 cells were inoculated in a well plate containing antibiotic-free medium at a density of 1 × 10^5^ cells/ml and cultured overnight. Lipofectamine™3000 (Life Technologies, Rockville, MA, USA) was transfected into OPTI-MEM-reduced serum medium (Gibco, USA) for 48 h according to production instructions. The influence of intervention was evaluated by real-time polymerase chain reaction (PCR).

### 2.5. Preparation and Analysis of RNA

Total RNA was extracted from cells and myocardial tissues with Trizol reagent (Invitrogen, USA) and reverse transcribed into cDNA with PrimeScript RT kit (Japanese Plateau City). Then, TB Green Premix Ex Taq II (Takara, Japan) was used to quantitatively amplify cDNA. Real-time PCR was performed in triplicate using the 6Flex application biology system. The expression of TAF9b was related to the expression of GAPDH gene. The expression of relative miR-199 was normalized to the expression of RNA (SnRNA) in U6. The amplification reaction conditions were pre-denaturation at 94°C for 2 min, denaturation at 94°C for 30 s, annealing at 49.3°C for 30 s, and extension at 72°C for 2 min, a total of 33 cycles. Finally, it was extended at 72°C for 5 min The primer sequence was as follows: MiR-199, F: 5′-AGAAGGCGATTGATACGAGTCA-3′, R: 5′-GGTCTCCCCAGTGTTCAGATA-3′. TAF9b, F: 5′-CGCAAGAGAAAATGGAGCCG-3′, R: 5′-CATCGTCCAGAATTGTAGTCACA-3′. Bcl-2, F: 5′-ATGCCTTTGTGGAACTATATGGC-3′, R: 5′-GGTATGCACCCAGAGTGATGC; Bax, F: 5′-TGAAGACAGGGGCCTTTTTG-3′, R: 5′-AATTCGCCGGAGACACTCG-3′; U6, F: 5′-GCTTCGGCAGCACATATACTAAAAT-3′, R: 5′-CGCTTCAGAATTTGCGTGTCAT-3′; GAPDH, F: 5′-CGCTCTCTGCTCCTCCTGTTC-3′, R: 5′-ATCCGTTGACTCCGACCTTCAC-3′. The PCR product was analyzed by ABI PRISM 7300 sequence detection systems (Applied Biosystems, Foster City, CA, USA). The expression of the target gene was calculated by 2^−△△CT^ method.

### 2.6. Dual-Luciferase Reporter Assay

The fragment of TAF9b mRNA containing miR-195 binding sites was inserted into the psiCHECK-2 luciferase reporter vector (Promega, Madison, WI, USA). The mutant plasmids were known as TAF9b-Mut. The abovementioned plasmid was transfected into cells containing NC mimics or miR-199 mimics by Lipofectamine 2000.48 h after transfection, the luciferase activities were measured using the dual-luciferase reporter assay system (Promega). Follow the instructions of the technical manual for the dual-luciferase reporter gene test kit. The internal reference of psiCHECK2 vector was firefly luciferase activity. The expression of psicheck2-TAF9B-3 UTR WT and psicheck2-TAF9B-3 UTRMUT were controls. Fluorescence intensity was detected 24 h after transfection. The ratio of the luminescence intensity of sea cucumber luciferase to that of firefly luciferase is the binding force of miR-199 and TAF9b.

### 2.7. ELISA Assay

The activity of superoxide dismutase 1 (SOD), malondialdehyde (MDA), lactate dehydrogenase (LDH), tumor necrosis factor-*α* (TNF-*α*), interleukin-1*β* (IL-1*β* cells), and interleukin-6 (IL-6) was measured using commercial kits from Nanjing Jiancheng Institute of Biological Engineering.

### 2.8. Flow Cytometry

To detect the apoptotic rate, the cells were seeded in 12-well plates at the seeding density of 3 × 10^5^/well and cultured for 48 h. Thereafter, the cells were washed twice with PBS, resuspended in binding buffer, and then added with Annexin V-FITC and propidium iodide (PI) in the dark for 15 min at 37°C. The cell apoptosis rate was analyzed by flow cytometry within 1 h.

### 2.9. TUNEL Staining

TUNEL apoptosis detection kit (Alexa Fluor488; Yeasen, China) was used to detect nuclear fragmentation according to the regulations of the manufacturer. For TUNEL staining of AC16 s, the cells were washed with PBS and fixed with 4% paraformaldehyde. Tissue sections and cells were incubated with protease K for 5 min, permeability solution 0.1% and Triton X-100 in 4°C for 2 min. Rinse cells with PBS twice, 5 min each. TUNEL reaction solution (TdT + fluorescein labeled dUTP) was added, and incubated in a wet box at 37°C for 60 min in the dark. Wash cells with PBS for 3 times, 5 min each, and stained with Hoechst33342 (Beyotime Biotechnology, China). In fluorescent staining, the nuclei appear to be morphologically altered by blue fluorescence. Then, the apoptotic cells were observed under a fluorescence microscope (Nikon, Japan) and counted from five randomly selected regions by image J.

### 2.10. Western Blot

AC16 cells were collected after DOX treatment for 24 h. After the cells were treated with cell lysate, an appropriate amount of electrophoresis sample buffer was added. Afterward, the sample was heated in boiling water for 10 min, and then electrophoresis in 12% polyacrylamide gel was performed. The sample was blocked with 3% BSA for 2 h [25] at 37°C. Mouse anti-human Beclin-1 (Abcam, 1 : 1000, Cambridge, MA, USA), LC3B (Abcam, 1 : 1000) antibody, and mouse anti-human GAPDH (Abcam, 1 : 1000) were added overnight at 4°C and washed with PBST three times each time. The corresponding secondary antibody labeled with HRP was added, incubated at 37°C for 30 min, and washed with PBST three times for 15 min each time. The results were visualized by Odyssey Infrared Imaging System.

### 2.11. Statistical Analysis

All data were expressed as mean ± SD of at least three independent experiments. SPSS 22.0 software (SPSS Inc., Chicago, IL, USA) was implemented for statistical analysis. The difference between the two groups was tested by Student's *t*-test. Bonferroni posttest was performed following one-way ANOVA and was considered statistically significant.

## 3. Results

### 3.1. DOX-Induced Myocardial Cell Injury (AC16 Cells)

We used Adriamycin (0.5 *μ*m) to establish the myocardial cell injury model in vitro, and study the effects of Adriamycin on AC16 cells. The experimental results showed that the cell proliferation rate in the DOX-induced group was significantly lower than that in the control group (Figure 1(a)). We also detected the inflammatory factors in the two groups. The results revealed that TNF-*α*, IL-1*β*, and IL-6 in the DOX-induced group were evidently high (Figure 1(b)). Then, we detected LDH, SOD, and MDA in the two groups. The results revealed that the LDH and MDA in the DOX-induced group were high with low MDA (Figure 1(c)). We used flow cytometry to detect apoptosis in the two groups. The results showed that the apoptotic rate in the DOX-mediated group was evidently high (Figure 1(d)). We performed TUNEL staining, and the results revealed that the apoptotic rate and Bax of the DOX-mediated group were high (Figure 1(e)). On the contrary, Bcl-2 of the DOX-mediated group was low (Figure 1(f)). Finally, Beclin-1 and LC3B-II in the DOX-induced group were higher than those in the matched group (Figure 1(h)). Therefore, DOX could damage AC16 cells.

### 3.2. DOX Promotes miR-199 Expression

Our study unmasked that DOX could promote the expression of miR-199. miR-199 of cardiomyocytes in the control and DOX-induced groups was quantified. The results revealed that miR-199 of cardiomyocytes in the DOX-induced group was high (Figure 2(a)). In addition, miR-199 of cardiomyocytes in the DOX-mediated group (5 mg/kg) was higher than that in the matched group (Figure 2(b)). We further performed HE staining of DOX-induced myocardial injury in mice (Figure 2(c)). The results showed that the DOX-induced group had significantly increased myocardial cell damage compared with the control group. Therefore, DOX could promote miR-199 expression.

### 3.3. Overexpression of miR-199 Promotes Cardiotoxicity of DOX

Our study showed that overexpression of miR-199 could promote cardiotoxicity of DOX. First, miR-199 was divided into four groups induced with DOX. Each group of mimics-NC, miR-199 mimics, inhibitor-NC, and miR-199 inhibitor was prepared (Figure 3(a)). The results revealed that TNF-*α*, IL-1*β*, and IL-6 were overexpressed in the miR-199 mimic-transfected group (Figure 3(b)). Second, LDH, SOD, and MDA were detected, and we found that LDH and MDA were overexpressed in the miR-199 mimic group after transfection (Figure 3(c)). However, the expression of SOD in the miR-199 mimic group was low (Figure 3(c)). We used flow cytometry to detect apoptosis in each group and obtained the same results; the apoptotic rate of cells transfected with miR-199 mimics was the highest (Figure 3(d)). Then, we performed TUNEL staining to detect apoptosis in each group, and the results suggested that the apoptotic rate of cells transfected with miR-199 mimics was the highest (Figure 3(e)). The TUNEL staining results were consistent with the results of flow cytometry. We detected the expression of Bax and Bcl-2 in each group. The results displayed that Bax was overexpressed in the miR-199 mimic group after transfection (Figure 3(f)), and Bcl-2 expression was distinctly low in the miR-199 mimic group after transfection (Figure 3(g)). Finally, we concluded that the miR-199 mimic-transfected group was overexpressed (Figure 3(h)). Furthermore, the overexpression of miR-199 could promote the cardiotoxicity of DOX.

### 3.4. TAF9b Is a Target Gene Mediating the Regulatory Characteristics of miR-199

In our study, TAF9b is the target gene that mediates the regulatory characteristics of miR-199. The schematic diagram of the combination of miR-199 and TAF9b is shown in Figure 4(a). Luciferase reporter assay revealed that the fluorescence activity of the TAF9b-WT group reduced markedly, whereas no difference was found in the TAF9b-MUT group. This result indicated that TAF9b was the target of miR-199a. Subsequently, we detected TAF9b expression of cardiomyocytes in the control and DOX-mediated groups (0.5 *μ*M) at the cellular level. The results displayed that TAF9b expression of cardiomyocytes in the DOX-mediated group (0.5 *μ*M) was lower than that of the matched group (Figure 4(c)). In addition, we detected TAF9b expression of cardiomyocytes in the control and DOX-induced groups (0.5 *μ*M) at the animal level. The results revealed that TAF9b of cardiomyocytes in the DOX-induced group was low (Figure 4(d)). We also found that the knockdown of miR-199 could upregulate the expression of TAF9b at the cellular level (Figure 4(e)). Therefore, we concluded that TAF9b was the target gene that mediated the regulatory characteristics of miR-199.

### 3.5. Knockdown of TAF9b Reverses the Cardioprotective Effect of miR-199 Inhibitor

Our study showed that the knockout of TAF9b could reverse the protective effect of miR-199 inhibitor on the myocardium. The induction of DOX was divided into the following groups: inhibitor-NC group, miR-199 inhibitor group, si-NC group, and miR-199 inhibitor + si-TAF9b group. First, the expression of TAF9b was detected in each group. The results indicated that the expression of TAF9b was high in the miR-199 inhibitor group (Figures 5(a) and 5(b)). Second, cell activity was detected, and the results revealed that the level of cell activity was the highest in the miR-199 inhibitor group (Figure 5(c)). Third, inflammatory cytokines were decreased in the miR-199 inhibitor group (Figure 5(d)). Fourth, LDH, SOD, and MDA of each group were detected, and the results revealed that LDH, SOD, and MDA in the miR-199 inhibitor group decreased evidently (Figure 5(e)). Fifth, the expression of Bax and Bcl-2 in each group was detected. The results revealed that Bax in the miR-199 inhibitor group was decreased (Figure 5(f)), whereas Bcl-2 in the miR-199 inhibitor group was evidently increased (Figure 5(f)). Therefore, the knockout of TAF9b could reverse the protective effect of miR-199 inhibitor on the myocardium.

### 3.6. Overexpression of TAF9b Reverses Injury Mediated by miR-199

Our study showed that overexpression of TAF9b could reverse the myocardial injury of miR-199. DOX induction was divided into the following groups: mimics-NC group, miR-199 mimic group, vector-NC group, and miR-199 mimics + TAF9b group. First, we detected the apoptosis in each group by flow cytometry. The results suggested that the apoptotic rate in the miR-199 mimic + TAF9b group was lower than that in the miR-199 mimic group (Figures 6(a)-6(b)). Second, we used TUNEL staining to detect apoptosis in each group. The results revealed that the apoptotic rate in the miR-199 mimics + TAF9b group was evidently lower than that in the miR-199 mimic group (Figure 6(c)). Third, we detected the expression of Bax and Bcl-2 in each group. The results revealed that Bax in the miR-199 mimics + TAF9b group was evidently lower than that in the miR-199 mimic group (Figure 6(d)), and Bcl-2 in the miR-199 mimics + TAF9b group was distinctly lower than that in the miR-199 mimic group (Figure 6(e)). Finally, we detected autophagy-related proteins, including Beclin-1 and LC3B by western blot. The results showed that overexpression of miR-199 promoted the expression of Beclin-1 and LC3B compared with the control group. However, Beclin-1 and LC3B decreased in miR-199 mimics + TAF9b group (Figure 6(f)). Therefore, overexpression of TAF9b can reverse miR-199-mediated autophagy in cardiomyocytes.

## 4. Discussion

DOX is a widely used anticancer drug [35–37]. However, the clinical application of DOX is limited because of its potential to cause severe heart failure and degenerative cardiomyopathy in the elderly patients with previous heart disease [38,39]. Its cardiotoxicity limits its clinical treatment. Although several mechanisms of toxicity have been proposed [40–42], the mechanism of toxicity in other organs remains elusive, but the role of oxidative stress shows great potential as a mechanism of DOX-induced cardiotoxicity [43–45]. Some scholars have proposed the adverse outcome pathway (AOP) mechanism, but AOP is still in its infancy, which plays a little role in the establishment of complex toxicology. However, the tools of AOP can be used for toxicology and risk assessment in the future, as it can comply with the OECD guidelines [46]. Chemically mediated skin allergy, cholestasis, and liver-related diseases are examples of AOPs [47]. In addition, in 6 to 8-week-old C57BL/6N mice, the destruction of intestinal epithelial cells was the common cause of adverse reactions caused by DOX (20 mg/kg, i.p.), which led to the leakage of intestinal microorganism-related endotoxin and enhanced TLR4 signal. Immunotoxicity is caused by systemic inflammation and multiple-organ injury [48,49].

DOX can distinctly inhibit cell viability and cell respiration, induce cell morphological changes, and increase reactive oxygen species. Despite considerable evidence supporting the role of microRNAs (miRNAs) in dose-mediated myocardial injury, the definite pathogenesis remains unclear. miRNA-128-3p promotes oxidative stress by targeting Sirt1, which aggravates the damage mediated by oxidative stress to Dox [50]. Zhao et al. screened 18 differentially expressed microRNAs using the microRNA microarray analysis technique in rat heart tissue mediated by DOX [51]. The results displayed that DOX increased miR-140-5p. Liu et al. proposed that let-7f-2-3p regulated by lncRNA NEAT1 aggravated DOX-mediated cardiotoxicity by inhibiting the HAX-1 nuclear outlet [52]. Hanouskova et al. [53] reported that after DOX treatment, miR-34a and miR-130a expression evidently increased [54], whereas miR-502 expression decreased [55]. However, no change was found in miRNA expression associated with troponin T. A study on the changes of plasma miRNA expression in children mediated by DOX associated with markers of heart injury showed that plasma miR-499 and miR-29b enhanced after DOX induction [56]. MiR-15 b-5p might be involved in DOX-mediated cardiotoxicity by suppressing the Bmpr1a signaling pathway in cardiomyocytes [57].

Autophagy is also an adaptive response, but when the external stimulation is excessive, the uncontrolled autophagy may not maintain the homeostasis of cardiomyocytes [58]. The complex interaction between cardiomyocyte apoptosis and autophagy determines the degree of myocardial damage and apoptosis [59]. In this study, the role of apoptosis and autophagy in DOX-mediated myocardial injury was investigated through low-dose long-term DOX intervention.

In previous studies, the role of autophagy in DOX-mediated myocardial injury has been widely debated [60–63]. In our study, we found that the relative cell proliferation rate in the DOX induction group was evidently lower than that in the matched group; the inflammatory factors in the DOX induction group were higher; the LDH and MDA in the DOX induction group were evidently higher. In addition, we implemented TUNEL staining and found that the apoptotic rate in the DOX-induced group was higher than that of the matched group. Using flow cytometry, we found that the apoptotic rate and Bax in the DOX-mediated group were high, and Bcl-2 in the DOX-mediated group was lower than that in the matched group. Therefore, DOX could damage AC16 cells. We further discovered that DOX could promote the expression of miR-199, and overexpression of miR-199 could promote the cardiotoxicity of DOX. The expression of TAF9b in cardiomyocytes mediated by DOX (0.5 *μ*M) was low. However, at the cellular level, knockdown of miR-199 could upregulate the expression of TAF9b; therefore, TAF9b mediated the regulatory characteristics of miR-199. If the knockout of TAF9b could reverse the protective effect of miR-199 inhibitor on the myocardium, then the overexpression of TAF9b could reverse the effect of myocardial injury on miR-199. Li et al. found that miR-199 was associated with physiological myocardial hypertrophy in mice [64]. Moreover, Baumgarten et al. found that Twist1 modulated the activity of the ubiquitin-proteasome system in human end-stage dilated cardiomyopathy via miR-199 [65].

In this study, miR-199 could aggravate DOX-induced myocardial injury by targeting TAF9b through in vivo and in vitro experiments. This study is the first to report the relationship between miR-199 and TAF9b. It enriches the understanding of miRNA-mRNA regulatory interactions. However, further studies are needed before the clinical application of miR-199. In addition, the downstream regulatory mechanisms of TAF9B have not been fully elucidated.

## 5. Conclusion

In this study, we found that miR-199 aggravates apoptosis and regulates autophagy in DOX-mediated cardiotoxicity by targeting TAF9b, and miR-199 may be a potential target for the treatment of DOX-mediated cardiotoxicity.

## Figures and Tables

**Figure 1:** Cardiomyocytes (AC16 cells) was injured by DOX. (a) The cell proliferation rate in the DOX induction group was distinctly lower than that in the control group. (b) The levels of TNF-*α*, IL-1*β*, and IL-6 in the DOX induction group were obviously higher. (c) The LDH and MDA in the DOX induction group was higher than that in the control group, while SOD in the DOX induction group decreased relatively to the control group. (d) Cell apoptosis detection by flow cytometry. (e) Detection of apoptosis cells by TUNEL staining. (f-g) Apoptosis-related protein expression detection by qPCR. (h) Beclin-1 and LC3B expression detection by western blotting. ^*∗*^*P* < 0.05, ^*∗∗*^*P* < 0.01, and ^*∗∗∗*^*P* < 0.001.

**Figure 2:** DOX promotes the expression of miR-199. (a) Detection of miR-199 in DOX-mediated cell model. (b) Detection of miR-199 in DOX-mediated mice model. (c) The myocardial tissue injury was observed by HE staining. ^*∗*^*P* < 0.05 and ^*∗∗*^*P* < 0.01.

**Figure 3:** Overexpression of miR-199 promotes the DOX-mediated cardiotoxicity. (a) Detection of miR-199 expression level in AC16 cells model after different treatment. (b) Detection of TNF-*α*, IL-1*β*, and IL-6 after different treatment. (c) Detection of LDH, SOD, and MDA by ELISA method. (d) Cell apoptosis test by TUNEL staining. (e) Cell apoptosis test by flow cytometry. (f) & (g) Detection of mRNA levels of Bax and Bcl-2 by RT-qPCR. (h) Beclin-1 and LC3B detection by western blotting. ^*∗*^*P* < 0.05, ^*∗∗*^*P* < 0.01, and ^*∗∗∗*^*P* < 0.001. Magnification: 200x.

**Figure 4:** TAF9b binds to miR-199 as a target gene. (a) The schematic diagram of the combination of miR-199 and TAF9b. (b) Detection of TAF9b in DOX-mediated AC16 cell model. (c) Detection of TAF9b expression level in DOX-mediated mice model. (d) Detection of TAF9b expression level after different treatment by RT-qPCR. (e) Detection of TAF9b expression level after different treatment by RT-qPCR. ^*∗∗*^*P* < 0.01 and ^*∗∗∗*^*P* < 0.001.

**Figure 5:** Knockdown of TAF9b reverses the cardioprotective influence on miR-199 inhibitor. (a) Detection of TAF9b expression level. (b) Detection of TAF9b expression level in AC16 cells model after different treatment. (c) Cell viability test by CCK-8 method. (d) Detection of TNF-*α*, IL-1*β*, and IL-6 after different treatment. (e) Detection of the content of LDH, SOD, and MDA in DOX-mediated cell model by ELISA method. (f) Bax and Bcl-2 test by RT-qPCR. ^*∗*^*P* < 0.05, ^*∗∗*^*P* < 0.01, and ^*∗∗∗*^*P* < 0.001.

**Figure 6:** Overexpression of TAF9b reverses injury mediated by miR-199. (a) Transfection efficiency of TAF9b overexpressing plasmid. (b) Detection of AC16 cell apoptosis by flow cytometry. (c) AC16 cell apoptosis test by TUNEL staining. (d, e) Detection of mRNA level of Bax and Bcl-2 by RT-qPCR. (f) Beclin-1 and LC3B expression detection by western blotting. ^*∗*^*P* < 0.05, ^*∗∗*^*P* < 0.01, and ^*∗∗∗*^*P* < 0.001.

## Data Availability

The data used to support the findings of this study are available from the corresponding author upon request.
